RETRACTED

# Clinical Treatment and Prognostic Analysis of Patients with Aneurysmal Subarachnoid Hemorrhage

**DOI:** 10.1155/2021/1250334

**Published:** 2021-12-02

**Authors:** Xue Yang, Qiong Cheng, Yunfei Li, Zheng Zheng, Junpeng Liu, Zhenhua Zhao

**Affiliations:** ^1^Department of Neurology, Fujian Provincial Hospital, Fuzhou 350001, Fujian, China; ^2^Provincial Clinical Department of Fujian Medical University, Fuzhou 350001, Fujian, China

## Abstract

Subarachnoid hemorrhage (SAH) is a serious disease caused by blood flow into the subarachnoid space due to rupture of blood vessels. All diseases that cause intracranial hemorrhage are the cause of subarachnoid hemorrhage. Among them, due to the particularity of intracranial blood vessels, intracranial blood vessels are more prone to aneurysms than other parts. Therefore, the incidence of aneurysmal subarachnoid hemorrhage (aSAH) is extremely high. The purpose of this article is to study the clinical treatment and prognosis analysis of aSAH patients. This article first summarizes the current status of SAH research at home and abroad and summarizes its potential value and significance. On this basis, an in-depth study of the clinical treatment of aSAH patients has been carried out. The physiological mechanism and clinical general differences of aSAH were studied and analyzed. This article systematically describes the application of CTP in the treatment and prognosis analysis of aSAH patients. Then, it will use a comparative analysis method, interdisciplinary method, and other research forms to carry out experimental research on the theme of this article. Research shows that rebleeding and blood sodium are the main factors for cerebral ischemia caused by aSAH.

## 1. Introduction

aSAH is a common disease of cerebrovascular diseases, and its incidence is second only to cerebral thrombosis and hypertensive cerebral hemorrhage. According to relevant statistics, 85% of subarachnoid hemorrhage are caused by rupture and bleeding of intracranial aneurysm, which belongs to clinical acute and critical patients [1, 2]. According to investigations, the proportion of subarachnoid hemorrhage caused by aneurysm rupture is about 7/100,000 to 20/100,000. ASAH accounts for about a quarter of all brain death patients [3, 4].

In the study of subarachnoid hemorrhage, many experts and scholars at home and abroad have achieved good results. For example, NaidechA has studied neurogenic cardiac coma in response to physiological doses of dobutamine and millinon, a complication of subarachnoid hemorrhage [5]. Dong analyzed the protective effect of melatonin on SAH-induced early brain injury and its potential mechanism to study the clinical treatment of subarachnoid hemorrhage [6]. These studies provide a meaningful reference for the clinical treatment and prognosis of aSAH.

RETRACTED

This article aims to improve the cure rate of aSAH patients and analyze the clinical treatment and prognosis of aSAH. By scoring different levels of fluid delivered by patients, each index is scored, and finally, the regression analysis of the status of different groups is carried out to analyze the feasibility of the research content of this article.

## 2. Clinical Treatment and Prognosis Study of Patients with aSAH

### 2.1. Surgery-Related Prevention and Treatment

#### 2.1.1. Prevention and Surgery of sASH Rebleeding

Rebleeding and cerebral vasospasm (CVS) are two important factors that need to be considered in the treatment of aneurysm patients. In the past, the relationship between these two factors and the timing of surgery was controversial. Surgical treatment during cerebral vasospasm can aggravate cerebral vasospasm. Waiting for surgery after cerebral vasospasm is considered to increase the risk of rebleeding [7, 8]. In recent years, with the development of medicine, the treatment of endovascular diseases has gradually tended to mature, and the aSAH mortality rate has decreased significantly, but due to its poor treatment effect, scholars have more controversy about the treatment of aSAH. The current view advocates early surgical treatment to reduce the risk of rebleeding and better prevent cerebral vasospasm [9, 10].

#### 2.1.2. Clearance of Blood Clots in the Subarachnoid Space

Studies have shown that early removal of thrombus in the acute phase of the first bleeding can prevent CVS [11, 12]. The main methods of removing thrombus are mechanical removal during craniotomy, cerebrospinal fluid drainage, and the use of thrombolytic drugs. Mechanical removal during surgery is mainly to remove blood clots in the subarachnoid space as much as possible during surgery. Common methods of cerebrospinal fluid drainage are as follows:

1. Repeated lumbar puncture to draw bloody cerebrospinal fluid
2. Continuous drainage of brain cistern or ventricle
3. Continuous drainage of lumbar puncture catheter
4. Cisterna magna is placed in a tube for continuous drainage

The route of administration of thrombolytic drugs includes intrathecal injection in the cisterna magna and direct intrathecal injection. It can also be injected through cistern, ventricle, lumbar puncture, or large cistern tube. Commonly used drugs are t-PA and UK [13, 14].

To help prevent CVs, we should avoid tissue traction and injury, completely stop bleeding, clean the skull cavity before surgery, and apply a vasodilator around the aorta (usually, 0.3% papaverine, 1% procaine, sodium nitrope, etc.).

RETRACTED

### 2.2. Analysis of the Pathophysiological Mechanism of Poor Prognosis in SAH Patients

The cerebral artery carries about 20% of the body's blood flow, but the arterial wall is very thin, similar to veins the same size elsewhere in the body, no medial and outer membranes compared to other arteries; therefore, the incidence of aSAH is very high. When blood pressure surges for a variety of reasons, the aneurysm suddenly breaks up, causing blood to flow into the subarachnoid cavity of the brain, which increases the skull content and intracranial pressure, causing secondary CVS [15].

CVS is another important reason for the poor prognosis of SAH patients. CVS caused by SAH refers to the narrowing of blood vessels caused by contraction or damage of one or more large arteries. This stenosis can be seen in angiography or ultrasonography and can cause delayed ischemic nerve damage and even death in severe cases. Obviously, the amount of subarachnoid hemorrhage in the cistern is significantly related to the development of CVS. If there is no bleeding in the basal cistern within 4 days after SAH, the patient rarely develops vasospasm. The cause of CVS is not yet clear, and it may involve multiple mechanisms, including the vasoconstrictor effect of OxyHb, which is produced by red blood cell breakdown after bleeding. The reduction of vascular endothelial-derived NO content increases the endothelin content and enhances the sensitivity of blood vessels to endothelin.

### 2.3. Analysis of Differences in General Clinical Factors of aSAH

#### 2.3.1. Clinical Analysis of aSAH

The subjects of this study are patients over 18 years of age (it is difficult to collect data from patients under 18 years of age, so patients aged over 18 years were selected) who have been diagnosed as aSAH by CTA, DSA, or surgery in a certain place. A retrospective analysis of the relationship between the clinical observation indicators of aSAH and the prognosis of delayed cerebral ischemia was conducted to screen important related risk factors and early assessment of patient status. We followed an active preventive treatment, strengthened the monitoring of the operation period, responded to adverse reactions in a timely manner, and achieved the goal of improving the prognosis of patients.

*(1) Distribution of Aneurysms*. A total of 82 aneurysms were found in 73 patients. The patient has multiple unit aneurysms. Internal carotid aneurysms are the most common, followed by the anterior cerebral artery and the middle cerebral artery. The specific location is shown in Figure 1.

*(2) Comparison of Clinical Data among Different Groups*. There was a statistically significant difference in GCS scores between the delayed cerebral ischemia group and the nondelayed cerebral ischemia group. There were statistically significant differences in GCS, intraventricular hemorrhage, and rebleeding between the good prognosis group and the poor prognosis group (*P* < 0.05). Details are shown in Table 1.

RETRACTED

The GCS and WFNS scores at admission reflect the severity of the patient's condition at the time of admission, indicating that the severity of early brain injury determines the patient's prognosis. When an aneurysm hemorrhage invades the ventricle, it will interfere with the normal circulation of the patient's cerebrospinal fluid, increase the intracranial pressure, and cause secondary brain damage to the brain more easily and will worsen the patient's prognosis.

#### 2.3.2. Analysis of the Difference of aSAH General Factors

*(1) Correlation Analysis of aSAH, Gender, and Age*. Intracranial aneurysms tend to occur in middle-aged and elderly people, and the incidence of men and women is basically the same, which is different from the results of previous studies. Some researchers believe that the incidence of aneurysms will increase with age. This may be due to degenerative changes in blood vessels with age. Due to the interaction of many factors, the elasticity of the blood vessel wall is weakened, and the female patient enters menopause. When the level of estrogen drops, its protective effect on blood vessels will also decrease, resulting in increased fragility of the blood vessel wall.

*(2) The Relationship between aSAH and Hypertension*. Long-term hypertension increases various inflammatory factors and *c* response proteins in blood vessels and further increases the amount of lipoprotein and endothelin present in blood vessels. The inner lining of the arteries is thickened and stiffened by inflammation, even causing cerebrovascular stenosis or occlusion.

*(3) The Relationship between aSAH and Wills Ring Variation*. The circle of Willis is the first stage of the internal cranial collateral circulation. If an acute infarction occurs, compensation can be made to establish collaterals. Effective collateral circulation increases the blood supply in the ischemic penumbra area, slows down the infarct rate, and reduces the infarct size. The variability of the anterior communicating artery and the variability of the left and right anterior cerebral arteries in the infarct group were statistically significant, while the remaining variability was not statistically significant. The area of the complete Wills ring in the cerebral infarction group was smaller than that of the incomplete Wills ring. Also, the prognosis is good, which may be related to the higher compensatory ability of full Wills ring.

RETRACTED

### 2.4. Application of Whole Brain CTP in aSAH

#### 2.4.1. The Application of CT in aSAH Intracranial Structure Extraction

Computer tomography (CT) technology plays an important role in medical imaging. The specific operation process is shown in Figure 2.

The following details the intracranial structure extraction algorithm:

Step 1: extracting the skull area
This step uses power-rate conversion, and the height characteristics of the skull pixels are considered in the power-rate conversion. The expression is defined as follows:
  (1) $$\begin{array}{c} s=c\times {\left(\frac{i}{255.0}\right)}^{r}\times 255+b. \end{array}$$
Among them, *i* is the gray value of the input pixel and *s* is the gray value of the processed output pixel. In this section, the values of the three constants are *c* = 1.2, *b* = 11, and *r* = 6.13.
Step 2: extracting the cranial cavity boundary
In this step, a left-right sweep algorithm based on the threshold level is used, which is a linear spatial filter.
Step 3: obtaining the mask image in the cranial cavity
In this step, in order to reduce the noise, the median filter is used to remove the noise in the image, and the filter size is 7 × 7. We choose the median filter here because it is not sensitive to extreme values and can remove outliers without affecting the clarity of the image.
Step 4: splitting the image
The mask image is morphologically multiplied with the source image (as in formula (2)), and the final intracranial structure is obtained.
  (2) $$\begin{array}{c} B_{2}=B_{1}\cdot M_{1}. \end{array}$$

#### 2.4.2. Application of Whole Brain CTP in aSAH

*(1) Analysis of Complications of aSAH*. The destruction products of blood and red blood cells accumulated by SAH in the subarachnoid space are the direct factors leading to vasoconstriction. The physiological change of the case is the release of various vasoactive substances and inflammatory mediators, such as vasoconstriction substances and vasodilator substances. It also includes changes in the structure of vascular endothelial cells and the function of vascular smooth muscle. The blood activates various growth factors, leading to changes in the proliferation of vascular endothelial cells and increased permeability and infiltration of inflammatory cells. Many complications can occur after sail, including aneurysm rupture and bleeding, cerebral vasospasm, subacute or acute hydrocephalus, seizures, hyponatremia, arrhythmia, cardiac dysfunction, pulmonary edema, lower extremity venous thrombosis, and anemia. Among them, aneurysmal rupture and rebleeding, CVs, hydrocephalus, and hyponatremia have the greatest impact on the prognosis of SAH. With the continuous progress of diagnosis and treatment technology in medical institutions, the popularization of digital subtraction angiography (DSA) and computed tomography angiography (CTA), the continuous maturity and progress of neurosurgical technology and intravascular treatment technology, the diagnosis of subarachnoid hemorrhage, and the treatment of aneurysms have been well solved. The risk of early death due to rebleeding has been relatively effectively reduced, but the overall mortality is still as high as 30% and the disability rate is 50%. The most common complications are hydrocephalus and delayed cerebral vasospasm [7]. For the prevention and treatment of hydrocephalus, there is still no good solution at home and abroad because of the interaction of many factors and complex mechanism.

*(2) Whole Brain CTP with Complications after aSAH*. Whole brain CTP can assess the blood perfusion state of the brain tissue of aSAH patients and provide hemodynamic information. Although CTP has a certain false alarm rate, its extremely high sensitivity can provide excellent preliminary screening capabilities. Test results show that CTP can correctly diagnose 80% of DCI patients, but DSA shows that only 73% of patients have CVS. There are significant differences in the CBF value between the DCI group and the non-DCI group.

*(3) Whole Brain CTP Assessment of the Efficacy and Prognosis of aSAH Patients*. During the hospitalization of aSAH patients, CTP was reviewed multiple times to provide dynamic cerebral perfusion information to monitor the effect of the patient's medication or surgery. Combined with cerebral artery CTA examination, it can assess the degree of arterial and vascular damage caused by surgical aneurysm clipping and endovascular interventional treatment.

RETRACTED

## 3. Experimental Study on the Clinical Treatment and Prognosis of Patients with aSAH

### 3.1. Experimental Protocol

To make the experiment more scientific and effective, we performed an experimental investigation of the complete clinical case data from 59 aSAH patients in a given region. Patients were aged between 30 and 70 years, and the male–female ratio was 5–7 years to ensure the validity of the experimental data. This experiment divided the patients into three groups, and the metrics were compared and scored for each group. The results of the present study were treated by SPSS22.0 and SNK to analyze and compare the results. It uses mathematical statistics to analyze the final results.

### 3.2. Research Methods

#### 3.2.1. Comparative Analysis Method

In this trial, 59 patients were divided into three different groups according to Hunt–Hess for comparative analysis. The results obtained provide a reliable reference for the final research results of this article.

#### 3.2.2. Mathematical Statistics

In this experiment, mathematical statistics is used to make statistics and analysis on the research results of this article.

#### 3.2.3. Interdisciplinary Approach

This research combines pathology, biomolecular science, computer science and technology, and other disciplines to conduct a multifaceted research and analysis of aSAH. The data obtained provide theoretical support for the final research results of this article.

## 4. Clinical Treatment and Prognostic Experimental Analysis of Patients with aSAH

### 4.1. Different Fluid Volume and Prognostic Analysis

In order to make this experiment more scientific and effective, this experiment compares and analyzes the GOS scores between different liquid volume groups. The data obtained are shown in Table 2.

It can be seen from Figure 3 that the first-level patients died and the fifth-level patients can live normally. Except for the third group with a score of 3.43, the other two groups are all below 3. This indicates that the fatality rate and disability rate of aSAH are extremely high. Also, the statistical difference *P* in the three groups is greater than 0.05, and it can be seen that there is no statistical difference between the different liquid volumes.

### 4.2. Analysis of Regression Status in Different Groups

In order to further study and analyze this experiment, this experiment uses statistically different indicators as independent variables and DCI and prognosis as dependent variables for binary logistic regression analysis. The data obtained are shown in Table 3.

It can be seen from Figure 4 that NLR and GCS scores are independent risk factors for delayed cerebral ischemia. Rebleeding and blood sodium are independent risk factors leading to poor prognosis of patients. Surgical treatment can be effective to improve the patient's treatment prognosis, and the higher the HUNT grade of the patient, indicating that the patient will increase the risk of cerebral vasospasm and aneurysm rupture in bleeding, thus affecting the patient's prognosis. Clinicians need to strengthen the dynamic observation of patients' cerebral blood flow in order to detect early, prevent delayed cerebral ischemia, improve patient prognosis, and enhance the clinical efficacy of postoperative treatment.

## 5. Conclusions

This article aims to study the clinical treatment and prognosis of aSAH patients. Through the analysis of the related surgical prevention and treatment of aSAH, the pathophysiological mechanism of the poor prognosis of aSAH patients is analyzed in depth. In this paper, the application of CT in the extraction of intracranial structures in aSAH and the application of whole brain CTP in aSAH have been systematically explained. The experiment in this paper proves that the mortality and disability rate of aSAH are very high. The statistical difference among the three groups was greater than 0.05, which showed that there was no statistical difference between different liquid volumes. NLR and GCS scores were independent risk factors for delayed cerebral ischemia. Rebleeding and blood sodium are independent risk factors for poor prognosis. Surgical treatment can effectively improve the prognosis of patients, and the higher the hunt level, the higher the risk of cerebral vasospasm and aneurysm rupture. There are many prognostic factors affecting the treatment in aSAH patients, including the gender and severity of the patient itself. Clinical measures should be taken according to the patient's relevant prognostic risk factors to improve the patient prognosis.

RETRACTED

## Figures and Tables

**Figure 1:** Distribution of aneurysms.

**Figure 2:** Intracranial structure extraction algorithm framework.

**Figure 3:** Comparison of GOS scores between different fluid volume groups.

**Figure 4:** Different group regression status analysis.

**Table 1:** Comparison of clinical data between different groups.

		Number of cases	Percentages (%)	*P*_1_ value	*P*_2_ value
Level of consciousness	Wide awake	40	54.8	0.7	0.12
	Lethargy	15	20.5		
	Hazy	5	6.8		
	Restlessness	3	4.1		
	Light coma	7	9.6		
	Deep coma	3	4.1		

GCS score	3–8	11	13.7	0.03	0.02
	9–13	12	16.4		
	14–15	50	68.5		

**Table 2:** Comparison of GOS scores between different fluid volume groups.

	1000–2500	2500–3500	3500–5500	*F*	*P*
Group 1	5.00	4.86	4.33	2.91	0.07
Group 2	4.60	4.38	3.80	1.16	0.33
Group 3	5.00	3.40	2.50	3.43	0.10

**Table 3:** Different group regression status analysis.

	OR value	95% CI	*P* value
NLR	1.628	0.203	0.001
GCS	0.680	0.482	0.034
Bleeding again	9.687	0.174	0.028
Blood sodium	0.792	0.648	0.024

## Data Availability

The data underlying the results presented in the study are available within the manuscript.
